RETRACTED

# INPP1 up‐regulation by miR‐27a contributes to the growth, migration and invasion of human cervical cancer

**DOI:** 10.1111/jcmm.14644

**Published:** 2019-09-26

**Authors:** Pu Li, Qiaoge Zhang, Hua Tang

**Affiliations:** ^1^ Tianjin Central Obstetrics and Gynecology Hospital Reproductive Medical Center Tianjin China; ^2^ Tianjin Life Science Research Center and Department of Pathogen School of Basic Medical Sciences Tianjin Medical University Tianjin China

**Keywords:** cervical cancer (CC), INPP1, miR‐27a

## Abstract

Inositol polyphosphate‐1‐phosphatase (INPP1) is an enzyme that is responsible for glycolysis and lipid metabolism. Here, we discovered that INPP1 expression was up‐regulated in CC tissues compared to that in adjacent normal tissues by RT‐qPCR. Inositol polyphosphate‐1‐phosphatase overexpression promoted and INPP1 knockdown suppressed cell viability, cellular migration/invasion and EMT in CC cells. To explore the mechanism of dysregulation, INPP1 was predicted to be a target of miR‐27a, and a pmiRGLO dual‐luciferase reporter assay showed that miR‐27a bound to the 3′ UTR of INPP1. RT‐qPCR revealed that miR‐27a was also up‐regulated and had a positive correlation with INPP1 expression in CC tissues. Furthermore, shR‐INPP1 could favour the malignant phenotype reversion induced by miR‐27a, suggesting that miR‐27a up‐regulates INPP1 to promote tumorigenic activities. Altogether, our findings show that the up‐regulation of INPP1 by miR‐27a contributes to tumorigenic activities and may provide a potential biomarker for CC.

## 1 INTRODUCTION

Cervical cancer (CC) is the third most common leading cause of cancer death among females in developing countries.^1^ More than 274 000 individuals die each year.^2^ In China, approximately 98 900 new cases were diagnosed in 2015, which accounted for 18.7% of the global incidence.^3^ Additionally, 30% of patients were <44 years old.^4^ Reportedly, the 5‐year survival rates for locally advanced CC vary as follows: 58% for stage IIB, 35% for IIIA, 32% for IIIB and 16% for stage IVA.^5^ Therefore, it is urgent to identify novel molecular markers to improve the early diagnosis rate of CC and to develop an effective treatment strategy.

Inositol polyphosphate‐1‐phosphatase (INPP1) is an enzyme that dephosphorylates free polyphosphorylated inositols,^6^ key molecules involved in phosphatidylinositol signalling pathways.^7^ Presently, it has been reported that INPP1 is up‐regulated in human colorectal cancer.^8^ Daniel et al^9^ also found that INPP1 is highly expressed in aggressive melanoma, prostate, ovarian and breast cancer cells to promote migration and invasion; this finding suggests that INPP1 may function as an oncogene. However, the role of INPP1 in CC is still unclear.

RETRACTED

MicroRNAs (miRNAs) are small non‐coding RNAs that can bind to the 3′ UTR of target mRNAs, resulting in translational repression or degradation to regulate a wide range of physiological and pathological processes.^10^, ^11^, ^12^ Recent findings demonstrate that miRNA also binds to the 3′ UTR of mRNAs to raise the expression levels of their target genes.^13^, ^14^, ^15^ Furthermore, accumulating evidence has indicated that the miRNA profiles were differentially expressed in human cancerous tissues and adjacent normal tissues.^16^, ^17^ The dysregulated miRNAs may function as tumour suppressors or oncogenes,^18^ which present diagnostic and prognostic values in clinical applications.^19^, ^20^ miR‐27a was found to be up‐regulated and to promote malignancy in non–small‐cell lung cancer, breast cancer, prostate cancer, liver cancer, CC, etc.^21^, ^22^, ^23^, ^24^, ^25^

In this report, we show that INPP1 is up‐regulated in CC tissues compared with the levels in adjacent normal tissues. Inositol polyphosphate‐1‐phosphatase promoted cell proliferation and invasion/migration. miR‐27a bound to the 3′ UTR of INPP1 to increase the expression in CC cells. Rescue experiments indicated that INPP1 is a functional target gene of miR‐27a. Overall, our present work proved that miR‐27a promotes INPP1 expression to contribute to the malignant properties of CC cells, which may serve as biomarkers for the diagnosis of CC.

## 2 MATERIALS AND METHODS

### 2.1 Human cervical cancer tissue specimens and cell lines

Twenty human CC tissues and adjacent normal tissues were obtained from the Tianjin Central Hospital of Obstetrics and Gynecology, China. Written informed consent was obtained from each patient, and ethics approval for this work was granted by the Ethics Committee of Tianjin Central Hospital of Obstetrics and Gynecology. The cervical samples were verified and classified by pathologists. The human CC cell lines HeLa and SiHa were cultured in RPMI 1640 medium containing 10% heat‐inactivated foetal bovine serum (FBS), 100 IU/mL penicillin and 100 μg/mL streptomycin. C33A was cultured in DMEM. All cells were incubated in a humidified atmosphere at 37°C with 5% CO_2_.

### 2.2 Plasmid construction

The miR‐27a precursor was cloned from the genome by PCR and was inserted into the pcDNA3 vector by BamHI/EcoRI digestion. Small interfering RNAs against miR‐27a (ASO‐miR‐27a) were synthesized by GenePharma. The wild‐type INPP1 3′ UTR including the target site of miR‐27a and a mutant containing a mutation in the miR‐27a target site were cloned into the pmiRGLO vector (Promega) using PmeI/XbaI digestion. The INPP1 cDNA was cloned from the mRNA by PCR and was inserted into the pcDNA3‐Flag vector using BamHI/XbaI digestion, thus generating pcDNA3‐Flag/INPP1 (pINPP1). Two strands were annealed and cloned into the vector pSilencer 2.1‐U6 neo (Ambion) using BamHI/HindIII digestion to construct the INPP1 shRNA expression plasmid pSilencer/shR‐INPP1 (pshR‐INPP1). The sequences of the primers used are listed in Table 1.

RETRACTED

**Table 1:** Sequences of the primers used in this study

Name	Sequence (5′‐3′)
pri‐miR‐27a‐S‐XhoI	CGCGGATCCACCCTGAGCTCTGCCACCG
pri‐miR‐27a‐AS‐EcoRI	CGGAATTCGCAGCAGGATGGCAGGCAGAC
ASO‐miR‐27a	GCGGAACUUAGCCACUGUGAA
ASO‐NC	CAGUACUUUUGUGUAGUACAA
miR‐27a‐RT	GTCGTATCCAGTGCAGGGTCCGAGGTATTCGCACTGGATACGACGCGGAAC
miR‐27a‐Fwd	TGCGGTTCACAGTGGCTAAG
U6‐RT	GTCGTATCCAGTGCAGGGTCCGAGGTGCACTGGATACGACAAAATATGG
U6‐Fwd	TGCGGGTGCTCGCTTCGGCAGC
Reverse	CCAGTGCAGGGTCCGAGGT
INPP1‐S‐BamHI	CAGGGATCCATGTCAGATATCCTCCGGGAG
INPP1‐AS‐XhoI	GCTCACCTCGAGCTAGGTATGCGTCTCTGCAGG
pmiRGLO‐INPP1‐3′UTR Top	AAACTAGCGGCCGCTAGTACCTGTATAAACTGAACTGTGAT
pmiRGLO‐INPP1‐3′UTR Bot	CTAGATCACAGTTCAGTTTATACAGGTACTAGCGGCCGCTAGTTT
pmiRGLO‐INPP1‐3′UTR‐MUT Top	AAACTAGCGGCCGCTAGTACCTGTATAAACTGATGACACTT
pmiRGLO‐INPP1‐3′UTR‐MUT Bot	CTAGAAGTGTCATCAGTTTATACAGGTACTAGCGGCCGCTAGTTT
INPP1‐qPCR‐Fwd	GCCTCGTTGACATTTACA
INPP1‐qPCR‐Rev	CAAGCCCTGTTTCTGGAT
β‐Actin‐qPCR‐Fwd	CGTGACATTAAGGAGAAGCTG
β‐Actin‐qPCR‐Rev	CTAGAAGCATTTGCGGTGGAC
shR‐INPP1‐Top	GATCCGCAAAGTCCTCAATGGTAACACTCGAGTGTTACCATTGAGGACTTTGCTTTTTGA
shR‐INPP1‐Bot	AGCTTCAAAAAGCAAAGTCCTCAATGGTAACACTCGAGTGTTACCATTGAGGACTTTGCG

### 2.3 RNA extraction and real‐time PCR

RNA from patient tissues was extracted by the miRcute miRNA Isolation Kit (Tiangen Biotech) according to the manufacturer's instructions. TRIzol reagent (Invitrogen) was used to isolate the total RNA from CC cells. Then, reverse transcriptase‐polymerase chain reaction (RT‐PCR) methods were used for cDNA synthesis with Moloney murine leukaemia virus (M‐MLV) reverse transcriptase (Promega). A SYBR Premix Ex Taq II Kit (Takara) was used for qPCR in a Thermal Cycler Dice™ Real Time System III (TaKaRa). β‐Actin or U6 snRNA was used as an internal control. The relative transcript‐level fold‐change was calculated using the 2^−∆∆Ct^ method.^26^

### 2.4 Western blot analysis

The protein samples were obtained by using radioimmunoprecipitation assay (RIPA) lysis buffer to lyse the cells for almost 30 minutes at 4°C. The primary antibodies used in the Western blot assay are as follows: (a) rabbit anti‐GAPDH (Tianjin Saier Biotech; 1:2000), (b) rabbit anti‐INPP1 (Abcam, 1:1000), (c) rabbit anti–E‐cadherin (Tianjin Saier Biotech; 1:1000) and (d) rabbit anti‐vimentin (Tianjin Saier Biotech; 1:1000). Anti‐rabbit IgG‐HRP secondary antibodies were also used for Western blotting. Lab Works™ Image Acquisition and Analysis Software (UVP) was used for the quantification of the bands in the form of grey intensities.

RETRACTED

### 2.5 Luciferase reporter assays

HeLa (4 × 10^4^ cells/well) or C33A (5 × 10^4^ cells/well) cells were inoculated into 48‐well plates. After 16 hours, 0.5 μg of pri‐miR‐27a, ASO‐miR‐27a or the controls and 0.5 μg of reporter vector pmiRGLO‐INPP1‐3′ UTR/mut were cotransfected using Lipofectamine 2000 reagent (Invitrogen). After 48 hours of transfection, the cells were lysed by the Dual‐Luciferase Reporter Assay System (Promega).

### 2.6 Cell viability assay and colony formation assay

HeLa (8 × 10^4^ cells/well), SiHa (1 × 10^5^ cells/well) and C33A (1 × 10^5^ cells/well) cells were inoculated into 24‐well plates. After 16‐18 hours, 1 μg of the plasmids was transfected using Lipofectamine 2000 reagent (Invitrogen). After 24 hours of transfection, the cells were digested with 0.01% trypsin and counted by a haemocytometer. HeLa (2 × 10^3^ cells/well), SiHa (3 × 10^3^ cells/well) and C33A (5 × 10^3^ cells/well) cells were inoculated into 96‐well plates to detect the cell viabilities by an MTT assay. HeLa (2 × 10^2^ cells/well), SiHa (3 × 10^2^ cells/well) and C33A (3 × 10^2^ cells/well) cells were seeded into 12‐well plates to detect the colony formation rate. The details were described previously.^27^

### 2.7 Wound healing and cell invasion assays

For the wound healing assay, the movement of cells into the scraped area was measured to determine cell migration at 0, 48 and 72 hours as described by Ref. 25 For the invasion assays, the cells at the lower surface of the filter were counted as described previously.^28^

### 2.8 Statistical analyses

The significant differences between the sample means obtained from the three independent experiments were analysed using two‐tailed Student's *t* tests. Multiple group comparisons were performed by two‐way analysis of variance (ANOVA). Pearson's correlation was used to assess the association between two factors. *P* ≤ .05 was considered statistically significant.

## 3 RESULTS

### 3.1 INPP1 is up‐regulated in cervical cancer tissues

To identify the role of INPP1 in CC, RT‐qPCR was used to examine the INPP1 expression levels in 20 pairs of CC tissues and their corresponding adjacent normal tissues. As shown in Figure 1A, the level of INPP1 mRNA was higher in the CC tissues than the levels in the normal tissues. The mean expression of INPP1 was increased by approximately fourfold (Figure 1B). Thus, INPP1 was up‐regulated in CC.

**Figure 1:** High expression of INPP1 in CC tissues. A, Twenty pairs of tumour tissues and their adjacent normal tissues from 20 patients were assayed by qRT‐PCR separately. The data were normalized to β‐actin, and the INPP1 expression in normal tissues was arbitrarily defined as 100%. B, The mean expression of INPP1 in tumour tissues and adjacent normal tissues is shown. The INPP1 expression in normal tissues was arbitrarily defined as 100%, and the data are the mean ± SD of 20 samples (***: *P* < .001)

RETRACTED

### 3.2 INPP1 promotes oncogenic activity in cervical cancer cells

To assess the role of INPP1 in CC, we constructed an INPP1 overexpression plasmid, pcDNA3‐Flag/INPP1 (pINPP1) and a knockdown plasmid, pSilencer/shR‐INPP1 (pshR‐INPP1). First, we validated the effects of these plasmids at the mRNA and protein levels by RT‐qPCR and Western blotting (Figure 2A). Next, to determine whether INPP1 influences the cell viability, MTT assays were used, and we suggested that INPP1 overexpression promoted cell viability, while INPP1 knockdown repressed the cell viability of HeLa and C33A cells (Figure 2B). Moreover, colony formation assays were performed to explore the effect of INPP1 on cell growth in HeLa and C33A cells. As shown in Figure 2C, compared with that in the control group, the colony formation rate was increased by approximately twofold in the pINPP1 group and was decreased by approximately 50% in the pshR‐INPP1 group in HeLa and C33A cells, respectively. To determine whether INPP1 affects the mobility of CC cells, wound healing assays and transwell assays were used to examine the migration and invasion capacity. When INPP1 was overexpressed, the rates of migration and invasion were significantly increased by 1.5‐fold and 1.8‐fold, respectively, whereas they were significantly reduced by approximately 40% and 47%, respectively, when INPP1 was knocked down in HeLa cells (Figure 2D,E). Similar results were observed in C33A cells (Figure 2D,E). To determine the mechanisms behind the effects of INPP1 on cell mobility, epithelial‐mesenchymal transition (EMT) markers were detected by Western blot. As expected, compared with the protein expression in the control groups, pINPP1 promoted vimentin protein expression and suppressed E‐cadherin protein expression, and pshR‐INPP1 suppressed vimentin protein expression and promoted E‐cadherin protein expression (Figure 2F); this finding indicates that INPP1 was able to promote EMT in HeLa and C33A cells. We also obtained similar results in SiHa cells (Figure S1). Altogether, these results indicate that INPP1 may function as an oncogene in CC cells.

**Figure 2:** INPP1 functions as an oncogene in CC cells. A, HeLa and C33A cells were transfected with the overexpression plasmid pINPP1 or with the knockdown plasmid pshR‐INPP1. Forty‐eight hours after transfection, RT‐qPCR (left) and Western blots (right) were used to examine the expression levels of INPP1. B, MTT assays were performed to examine the cell viability at 24, 48 or 72 h after transfection. C, Colony formation assays were used to evaluate the cell growth. HeLa and C33A cells were grown for 14 d, and the colony formation rate was calculated. D, Twenty‐four hours after transfection, HeLa and C33A cells that were resuspended in 200 μL serum‐free medium were seeded into inserts and were incubated for 60 h to examine the invasion abilities. After staining with crystal violet, the cells at the lower surface of the membrane were counted under a light microscope at five random fields. E, Wound healing assays were used to reveal the effect of INPP1 on the cell mobility. F, EMT‐associated markers were assessed by Western blots (*: *P* < .05, **: *P* < .01, ***: *P* < .001)

RETRACTED

### 3.3 miR‐27a targets and up‐regulates INPP1 expression

To study the potential mechanisms underlying the dysregulation of INPP1, we investigated the effect of miRNA on INPP1 expression. Bioinformatics analysis (http://www.targetscan.org/vert_71/) was used to predict the candidate miRNAs that regulate INPP1. miR‐27a was chosen for further studies because the INPP1 3′ UTR contains a miR‐27a target site, and miR‐27a has been reported to promote the malignancy of CC cells. RT‐qPCR was performed to detect the expression level of miR‐27a in the 20 pairs of tissues that had been used to measure the INPP1 mRNA levels. The results showed that miR‐27a was up‐regulated in these CC tissues compared with that in the adjacent normal cervical tissues (Figure 3A). The mean expression of miR‐27a was increased by approximately 14‐fold (Figure 3B). Furthermore, miR‐27a also displayed a positive correlation with INPP1 (Figure 3C). To alter the miR‐27a expression level, the miR‐27a expression plasmid pri‐miR‐27a and the antisense oligonucleotide ASO‐miR‐27a were used to overexpress or block the expression of miR‐27a in CC cells. After the transfection efficiency of pri‐miR‐27a and ASO‐miR‐27a was confirmed (Figure 3D), we examined the INPP1 mRNA and protein levels by RT‐qPCR and Western blotting after the alteration of miR‐27a levels in HeLa and C33A cells. As shown in Figure 3E,F, pri‐miR‐27a increased, while ASO‐miR‐27a decreased, the expression of INPP1. To further determine whether INPP1 was a direct target of miR‐27a, the 3′ UTR of INPP1 that contained the miR‐27a binding site or mutant site was cloned into a pmiRGLO Dual‐Luciferase miRNA Target Expression Vector to generate the pmiRGLO‐INPP1‐3′ UTR/mut vector (Figure 3G). The luciferase activities were decreased when pmiRGLO‐INPP1‐3′ UTR and pri‐miR‐27a were cotransfected, whereas cotransfection with ASO‐miR‐27a caused an increase in the luciferase activity compared with that in the control group. In contrast, the mutation of the miR‐27a binding site in the INPP1 3′ UTR abolished the effect of both pri‐miR‐27a and ASO‐miR‐27a on the luciferase activities in HeLa cells (Figure 3H). These results indicate that INPP1 is up‐regulated by miR‐27a at the post‐transcriptional level in CC cells.

RETRACTED

**Figure 3:** INPP1 is directly targeted by miR‐27a. A, The relative expression level of miR‐27a in 20 paired cervical tissues was determined using RT‐qPCR. U6 snRNA was used for normalization. B, The mean expression of miR‐27a in tumour tissues and normal tissues is shown. C, Pearson's correlation analysis indicated a positive correlation between the expression of miR‐27a and INPP1 (*r* = .5008, *P* < .05). D, RT‐qPCR was used to examine the effectiveness of the pri‐miR‐27a plasmid and the antisense oligonucleotide ASO‐miR‐27a. E and F, HeLa and C33A cells were transfected with pri‐miR‐27a, the control plasmid pcDNA3 or ASO‐miR‐27a and the oligonucleotide control ASO‐NC. After 48 h of transfection, the relative INPP1 mRNA (E) and protein (F) levels were tested by RT‐qPCR and Western blots. G, The sequence alignment and schematic diagram of miR‐27a (mid) with the wild‐type (top) and mutated (bottom) 3′ UTR of INPP1 are shown. The arrows indicate the mutational nucleotides. H, The luciferase activity was measured 48 h post‐transfection with pcDNA3/pri‐miR‐27a or ASO‐miR‐27a in HeLa and C33A cells along with the pmiRGLO‐INPP1‐3′ UTR or mut. All data represent the mean ± SD of three independent experiments. (*: *P* < .05, **: *P* < .01, ***: *P* < .001, #: no statistically significant difference)

### 3.4 Knockdown of INPP1 abolishes the malignant phenotype induced by miR‐27a in cervical cancer cells

To verify that INPP1 indeed acts as the functional target of miR‐27a, “rescue” experiments were performed. pri‐miR‐27a and pshR‐INPP1 were cotransfected into HeLa, C33A and SiHa cells. As expected, the down‐regulation of INPP1 abolished the promoting effects of miR‐27a on cell viability (Figure 4A, Figure S2A), growth (Figure 4B, Figure S2B), invasion (Figure 4C, Figure S2C) and migration (Figure 4D, Figure S2D). Furthermore, the abnormal expression of EMT markers caused by miR‐27a was also restored to normal levels after INPP1 knockdown (Figure 4E). Taken together, these data suggest that INPP1 is a functional target of miR‐27a.

**Figure 4:** Knockdown of INPP1 abrogates the effects induced by miR‐27a in CC cells. HeLa and C33A cells were cotransfected with pri‐miR‐27a or pshR‐INPP1. An MTT assay (A), a colony formation assay (B), a transwell invasion assay (C) and a wound healing assay (D) were performed to analyse whether INPP1 knockdown could functionally rescue the miR‐27a–induced phenotype. E, EMT‐associated markers were measured by Western blots. (*: *P* < .05, **: *P* < .01, ***: *P* < .001)

RETRACTED

## 4 DISCUSSION

Previous studies have reported that INPP1 is up‐regulated in the vast majority of colorectal cancers.^8^ A recent report found that INPP1 is a highly expressed metabolic enzyme in aggressive ovarian and melanoma cancer cells and in primary human tumours, which drives cancer aggressiveness through regulating glycolytic metabolism and glucose‐derived LPA synthesis.^9^ Cancer cells have a notable preference to utilize aerobic glycolysis, rather than mitochondrial oxidative phosphorylation, for glucose‐dependent ATP production, which is thought to be the basis of tumour formation and growth.^29^ Thus, INPP1 attracted our attention.

In this study, we demonstrated that INPP1 was more highly expressed in CC tissues compared with that in adjacent normal tissues and that INPP1 facilitated the malignant behaviour of CC cells. Specifically, INPP1 overexpression significantly promoted cell viability, colony formation, migration and invasion, whereas shRNA‐mediated INPP1 silencing inhibited these oncogenic features. In addition, Western blot assays indicated that the expression of EMT markers, such as E‐cadherin and vimentin, was significantly modulated by INPP1. Thus, INPP1 may function as an oncogene in CC.

The dysregulation of miRNAs has been found to play key critical roles in up‐ or down‐regulating the expression of its target gene^30^ and may be a marker of progression in CC.^31^ To determine the potential epigenetic mechanism of INPP1 up‐regulation in CC, we investigated the regulation of miRNA on INPP1. First, bioinformatics was used to predict the miRNAs that target the 3′ UTR of INPP1, including miR‐27a. A previous report suggested that the expression of miR‐27a was significantly higher in cervical intraepithelial neoplasia (CIN) 2‐3 compared to that in CIN1 (*P* = .023) and in squamous cell carcinoma (SCC) compared to that in CIN2‐3 (*P* = .033).^32^, ^33^ Many investigations have indicated that miR‐27a is overexpressed in CC.^25^, ^34^, ^35^ The potential role of miR‐27a is similar to that of INPP1. Due to previous reports that miRNAs can bind to the 3′ UTR of their target transcripts and enhance their expression,^16^, ^17^ we explored whether miR‐27a exerts its role through binding to the 3′ UTR of INPP1 to increase its expression. Thus, we first applied a luciferase reporter assay to determine whether miR‐27a binds to the 3′ UTR of INPP1. The results indicated that miR‐27a binds to the 3′ UTR of INPP1 to enhance the luciferase activity in the luciferase reporter assay. Next, using a gain‐of‐function and loss‐of‐function procedure, we uncovered that miR‐27a enhanced the INPP1 expression at the mRNA and protein levels by Western blotting and RT‐qPCR. In addition, RT‐qPCR was used to examine the expression of miR‐27a and INPP1 in 20 pairs of CC tissues and their corresponding adjacent normal tissues; the results showed the up‐regulation of both miR‐27a and INPP1, which supports our finding that miR‐27a up‐regulated INPP1 expression. However, its detailed mechanism needs to be understood. To determine whether INPP1 is the functional target gene of miR‐27a, we designed a rescue experiment. The results verified that INPP1 decreased the ability of miR‐27a to promote CC cells. Together, our data demonstrate that the miR‐27a–mediated up‐regulation of INPP1 may promote the tumorigenic activities of CC cells, which indicates that miRNAs target and up‐regulate their target gene expression and may provide new insight into tumorigenesis in CC.

RETRACTED

In summary, our findings indicate that both INPP1 and miR‐27a are up‐regulated in CC and that miR‐27a binds to the 3′ UTR of INPP1 to increase the expression of INPP1. The overexpression of INPP1 promotes cell viability, colony formation, migration, invasion and EMT in CC cells and implies its potential role as a biomarker in CC.

## CONFLICT OF INTEREST

None declared.

## AUTHOR CONTRIBUTIONS

Pu Li conceived and designed the experiments; Pu Li and Qiaoge Zhang performed and analysed most of the experiments; Hua Tang contributed to the analyses of data; Pu Li and Qiaoge Zhang wrote the manuscript.
